The article "Study of aerobic and anaerobic bacterial profile of nosocomial infections and their antibiotic resistance in a referral center, Southwest Iran: A three year cross-sectional study" was retracted in 2025. Reasons: lack of ethics approval or compliance; missing or withdrawn patient consent; concerns about the welfare of human subjects.

# Study of aerobic and anaerobic bacterial profile of nosocomial infections and their antibiotic resistance in a referral center, Southwest Iran: A three year cross-sectional study

**DOI:** 10.1371/journal.pone.0259512

**Published:** 2021-11-09

**Authors:** Nazanin Ahmadkhosravi, Azar Dokht Khosravi, Aram Asareh Zadegan Dezfuli, Mohammad Hashemzadeh, Morteza Saki, Fatemeh Jahangiri Mehr, Farokh Izadpour

**Affiliations:** 1 Student Research Committee, Ahvaz Jundishapur University of Medical Sciences, Ahvaz, Iran; 2 Infectious and Tropical Diseases Research Center, Health Research Institute, Ahvaz Jundishapur University of Medical Sciences, Ahvaz, Iran; 3 Department of Microbiology, Faculty of Medicine, Ahvaz Jundishapur University of Medical Sciences, Ahvaz, Iran; 4 Iranian Study Group on Microbial Drug Resistance, Iran; 5 Pain Research Center, Health Research Institute, Ahvaz Jundishapur University of Medical Sciences, Ahvaz, Iran; 6 Microbiology Section of Medical Laboratory, Emam Khomeini Teaching Hospital, Ahvaz Jundishapur University of Medical Sciences, Ahvaz, Iran; School of Medicine, Tehran University of Medical Sciences, ISLAMIC REPUBLIC OF IRAN

## Abstract

**Background:**

The drug resistance is expected to be the most important challenge in infection control in Iran, where there is no local report or standard drug resistance monitoring system. Therefore, this study aimed to investigate the aerobic and anaerobic bacterial profile of nosocomial infections and their antibiotic resistance in Ahvaz, southwest Iran.

**Methodology:**

The gram-positive and gram-negative bacteria were identified on the basis of conventional culture and biochemical tests. The antibiotic resistance of the bacterial isolates against antibiotics was determined by the disk diffusion method.

**Results:**

Among total 1156 collected positive samples, *E*. *coli* and coagulase-negative staphylococci (CoNS) were the most frequent pathogenic gram negative bacteria (GNB) and gram positive bacteria (GPB) respectively. Drug susceptibility testing revealed that among GNB, *P*. *aeruginosa* was 100% resistant to amikacin, cefepime, ciprofloxacin and tetracycline. In the case of *E*. *coli*, the resistance rate was (98%) for trimethoprim sulfamethoxazole and cefepime. For GPB, *S*. *aureus* showed the highest resistance rates to amikacin (100%) and clindamycin (100%). In addition, CoNS strains showed a high level of resistance to doxycycline (100%), erythromycin (100%) and cefoxitin (97%). In *Bacteroeides fragilis* isolates, the highest resistance rate belonged to clindamycin (72%), and *Clostridium perfringens* strains showed high level of resistance to penicillin (46%).

The article "Study of aerobic and anaerobic bacterial profile of nosocomial infections and their antibiotic resistance in a referral center, Southwest Iran: A three year cross-sectional study" was retracted in 2025. Reasons: lack of ethics approval or compliance; missing or withdrawn patient consent; concerns about the welfare of human subjects.

**Conclusion:**

The results highlighted that there are distinct factors leading to antimicrobial resistance in Ahvaz, southwest Iran. The primary contributors to the resistance development, include poor surveillance of drug-resistant infections, poor quality of available antibiotics, clinical misuse, and the ease of access to antibiotics. Moreover, similar factors such as self-medication and the lack of regulation on medication imports play a role in antibiotic resistance in the region.

## Introduction

Antimicrobial resistance (AMR) has become a global concern and can cross international boundaries and spread between continents [1]. AMR has been estimated to be responsible for 10 million people deaths per year worldwide and severely affects low/middle-income countries directly or indirectly [2]. The World Health Organization (WHO) called the Eastern Mediterranean Region, one of the regions with the weakest performance in combating AMR due to the lack of national action plans and programs for infection control and patient safety, as well as for poor awareness, fragmented information systems, inadequate monitoring and surveillance, weak laboratory capacity, inappropriate prescription, and counterfeit drugs and medicines [3]. In the category of AMR in bacteria, antimicrobial resistance threat is of paramount significance [4]. AMR impairs the human immune system ability to combat infectious diseases and contributes to different complications in vulnerable patients with underlying diseases. As the effectiveness of antibiotics is declining owing to the persistence of AMR, physicians have to use last-resort classes of medicine that are always unavailable in developing countries. Such medicines are highly expensive and have varied side effects [5]. I did not understand the meaning.

Iran is a country with a high rate of antibiotics consumption [2]. One of the most important reasons for AMR is the inappropriate and irrational use of antibiotics for therapeutic and nontherapeutic applications in hospitals. This behavior is mostly rooted in the absence of national guidelines for prescription and stem from the lack of uncontrolled and over-the-counter sale of medicines, particularly antimicrobials [6]. Overuse and over prescription of these agents are a long-term concern for Iran’s health system. Researchers have long time ago been warned of the excess use of antimicrobials and the resultant AMR as a forthcoming challenge for the health system of Iran. Considering the available meta-analysis information, it is evident that the Iranian population as a serious concern are confronted with a high rate of AMR to the bacteria, including *Staphylococcus aureus* with resistance to methicillin (20.48% to 90%), and *Klebsiella pneumonia* with 96% and 77% resistance rate to ampicillin and co-trimoxazole respectively [2, 5]. The rate of multi-drug resistant (MDR) *Pseudomonas aeroginosa* was also estimated as 58% [7]. Migration of a large group of Afghan and Iraqi population to Iran, due to political unrests in these countries over the previous decades as well as illegal drug and human trafficking through the eastern borders with Pakistan and Afghanistan, has prejudiced the health system of the country [8]. Drug resistance in Iran is expected to be the most significant challenge as there is no local report or monitoring system for such resistance [9–12]. The present study was conducted to investigate the aerobic and anaerobic bacterial profile of nosocomial infections and to evaluate their antibiotic resistance in southwest Iran.

The article "Study of aerobic and anaerobic bacterial profile of nosocomial infections and their antibiotic resistance in a referral center, Southwest Iran: A three year cross-sectional study" was retracted in 2025. Reasons: lack of ethics approval or compliance; missing or withdrawn patient consent; concerns about the welfare of human subjects.

## Materials and methods

### Collection of specimens

This cross-sectional study was performed on all clinical samples received to the Microbiology laboratory of Imam Khomeini referral Hospital, Ahvaz, Iran, during a 3 year period from February 2018 to December 2020. The hospital serves as a referral center for the public health and infection control and management in Ahvaz city. The patients’ demographic information including age, sex, and specimen type and other related information, were retrieved from the registration book of the Microbiology laboratory. Patients with incomplete or missed data records were excluded. Collected samples were stored on ice and transported to the laboratory for testing, usually within 4 hours after sampling. The samples were immediately analyzed, on the day of collection. Anaerobic samples were collected in plastic containers and then inoculated in thioglycollate broth (Merck, Darmstadt, Germany) using a sterile inoculation loop. The broth media were incubated at 37°C for 24–48 h under aerobic conditions. Then the subculture was performed on blood agar enriched with 5% defibrinated sheep blood prepared from Bahar Afshan Company, Tehran, Iran. The blood agar plates were transferred to a candle jar and incubated at 37°C for 24–48 hours [13].

### Ethics approval and consent to participate

The study was approved by the Research Ethics Committee (REC) of the Ahvaz Jundishapur University of Medical Sciences (IR.AJUMS.REC.1399.386), Ahvaz, Iran, after submission of the preliminary proposal, and necessary permission for sample collection was granted. The study was accepted by the Imam Khomeini hospital data protection authority. After having read the information letter concerning the study, all respondents were asked for oral and written consent to participate. We emphasized that participation was voluntary and that patients could withdraw from the research at any time. This study does not use retrospective study of medical records or archived samples, and the samples were recorded directly by the researchers themselves.

The article "Study of aerobic and anaerobic bacterial profile of nosocomial infections and their antibiotic resistance in a referral center, Southwest Iran: A three year cross-sectional study" was retracted in 2025. Reasons: lack of ethics approval or compliance; missing or withdrawn patient consent; concerns about the welfare of human subjects.

### Aerobic microbial investigation

The collected samples including urine, pus, blood, ear discharge, eye swab, genital swab, sputum, and nasal swabs were processed in Microbiology laboratory by gram staining, and cultivation on appropriate culture media and incubated for 24 hrs at 37°C. Blood and MacConkey agars were used for cultivation of non-fastidious bacteria and Chocolate agar for fastidious bacteria. The grown colonies were then underwent necessary conventional identification procedure. The biochemical tests specified for Gram-positive bacteria (GPB) were as follows: catalase, coagulase, bacitracin, pyrrolidonyl arylamide (PYR), optochin test, bile solubility, and Novobiocin. For Gram-negative bacteria (GNB) the tests including serial biochemical reactions and fermentation of carbohydrates i.e. oxidase, catalase, triple sugar iron agar, citrate utilization test, urease, lysine iron agar, Sulphur indole motility, mannitol fermentation, and indole test were performed [13]. The blood samples were collected in standard trypticase soy broth bottle and directly incubated at 37^°^C. In the event of any indication of growth, like hemolysis, gas production, and turbidity, the sample was sub-cultured on an appropriate solid medium for further identification.

### Needs extensive changes

#### Anaerobic microbial investigation

A Gram-stain smear was used for cytology investigation and detection of bacterial presence in specimens. For the isolation of aerobic organisms, specimens were plated onto chocolate, sheep blood (5%) (Liofilchem) phenylethyl alcohol (PEA) (Hi Meia, India), and MacConkey agar (Liofilchem, Italy) plate. The plates were incubated at 37°C under 10% CO2 and examined at 24 hours and 48 hours later. Pre-reduced vitamin K enriched brucella blood agar; kanamycin-vancomycin laked blood agar (KVLB, Basal Medium is Brucella agar; Fluka Chmie AG CH-9471 Buchs, Switzerland), bacteroides bile esculin (BBE, Himedia Laboratories Pvt. Ltd, India) and (PEA) agar were inoculated for isolation of anaerobic organisms. The plate media were incubated under 80% N2, 10% CO2, 10% H2, and 0% O2 in anaerobic jar by using Anoxomat (MART microbiology B.V. The Netherlands) and these plates examined at 48, 72, and 96 hours. The primary inoculated thioglycolate broth (Merck Co., Germany) was incubated for 10 days and subcultured in 2 series of plates in the same way mentioned above. For enrichment and isolation of *C*. *perfringens*, a drop of syringe specimen was introduced into cooked meat broth media (Que Lab Inc) and incubated at 45°C for 4–6 hours. Thereafter, one loop of this incubated media was subcultured in sheep blood agar plate and incubated under anaerobic condition and examined after 24 and 48 hours. All isolated anaerobes were identified after conducting anaerobic tolerance test using biochemical tests such as catalase production, indole, and sugar fermentation (sucrose, arabinose, xylose, and rhamnose) as well as MID8 (Mast Identification 8, according to manufacturer company’s instructions) [13].

The article "Study of aerobic and anaerobic bacterial profile of nosocomial infections and their antibiotic resistance in a referral center, Southwest Iran: A three year cross-sectional study" was retracted in 2025. Reasons: lack of ethics approval or compliance; missing or withdrawn patient consent; concerns about the welfare of human subjects.

#### Antibiotic resistance AMR profiles

The AMR of the bacterial isolates to antibiotics was determined by the disk diffusion method according to the Clinical & Laboratory Standards Institute (CLSI) Guideline [14]. Accordingly, the isolates were classified as sensitive and resistant based on the diameter of the clearing zone. The antibiotic discs represented thirteen classes of antibiotics (MAST, Berkshire, UK) were as: chloramphenicol (Chloramphenicol), ciprofloxacin (Fluorinated quinolones), clindamycin (Lincosamides), gentamycin (Aminoglycosides), erythromycin (Macrolides), sulphamethoxazole/trimethoprim (Sulphonamides), tetracycline (Tetracyclines), vancomycin (Glycopeptides), Quinupristin-dalfopristin (streptogramins), cefoxitin (penicillinase-stable penicillins), nitrofurantoin (nitrofurantoin), rifampin (ansamycins), and linezolid (oxazolidinones). For antimicrobial drug susceptibility assay in Gram-negative anaerobic bacteria isolated from these infections, the Minimum Inhibitory Concentration (MIC) of imipenem, chloramphenicol, metronidazole, clindamycin, cefoxitin, and penicillin G (Sigma chemical Co. USA) was determined by the agar dilution method. MIC of penicillin, metronidazole, clindamycin, cefoxitin for Gram positive anaerobic bacteria were determined by Etest strip (AB biomerieux, Sweden) according to CLSI guideline for anaerobic susceptibility testing. The phenotype defined as multiple dug resistance (MDR), extremely drug resistant (XDR) and pandrug resistant (PDR) according to the International Expert proposal for Interim Standards Guidelines [14–16].

#### Quality control

American Type Culture Collection (ATCC) standard strains, including Staphylococcus *aureus* ATCC 25923, *Pseudomonas aeruginosa* ATCC 27853, and *E*. *coli* ATCC 25922, were used as quality controls for antibiotic resistance method.

## Results

### Dissemination of positive cultures/specimens

During the period of study, 90 out of 1246 samples yielded no growth, 860 aerobic bacteria and 296 anaerobic bacterial positive growth samples were collected from patients. Within a three-year investigation from 2018 to 2020, data were acquired from 420, 358, and 378 private and public healthcare facilities in southwest Iran, respectively. A total of 1156 bacteria were selected for the study from diverse clinical specimens (blood, urine, pus, and sputum). Most of the isolates were obtained from male patients (Table 1) and were detected in adults in the age range of 24–64 years (n = 421/1156; 36%), followed by the age group of 14–24 years (n = 504/1156; 43%). The least number of isolates were found in patients older than 64 years of age. Distribution of bacterial infections in clinical are shown in Table 2.

The article "Study of aerobic and anaerobic bacterial profile of nosocomial infections and their antibiotic resistance in a referral center, Southwest Iran: A three year cross-sectional study" was retracted in 2025. Reasons: lack of ethics approval or compliance; missing or withdrawn patient consent; concerns about the welfare of human subjects.

**Table 1:** Age and sex distribution of patients with bacterial isolates.

Age group (y) Sex	Total		
	Male N (%)	Female N (%)	Bacteria N (%)
< 5	8 (0.1)	22 (0.5)	30 (0.03)
5–14	62 (0.08)	110 (28%)	172 (0.2
14–24	368 (47%)	136 (35%)	504 (0.35)
24–64	321 (41%)	100 (25%)	421 (0.37)
> 64	11 (0.2)	18 (0.4)	29 (0.03)
Total	770 (66%)	386 (33%)	1156 (100)

**Table 2:** Distribution of sample type and bacterial isolates from a study of the burden of antimicrobial resistance at Imam Khomeini Hospital (2018–2020).

Specimen type												
Isolates	Urine	Body Fluids	Stool	Ear Swab	Eye swab	CSF	Blood	Sputum	Puss	Nasal swab	Genital swab	Total
*Streptococcus* spp.	-	6	-	10	-	-	25	15	6	-	-	62
*Micrococcus* spp.	-	-	-	-	-	-	6	6	-	-	-	12
*S*. *auraes*	15	7	-	10	5	-	58	2	-	30	-	127
*CoNS*	48	23	-	-	4	-	23	-	22	10	-	130
*Enterococcus* spp.	12	1	5	-	-	-	12	-	2	-	-	32
*Klebsiella* spp.	31	5	-	4	-	-	30	12	15	-	-	97
*E*. *coli*	74	20	21	3	2	-	55	-	18	-	-	193
*Pseudomonas*	18	2	-	8	1	-	15	10	8	-	-	62
*Enterobacter* spp.	14	-	-	-	-	-	12	4	6	-	-	36
*Acinetobacter* spp.	40	-	-	9	2	-	22	-	22	-	-	95
*P*. *mirabilis*	12	-	-	-	-	-	-	-	-	-	-	12
*Stenotrophomonas* spp.	-	-	-	-	-	-	1	-	-	-	-	1
*C*. *freundii*	-	-	-	-	-	-	1	-	-	-	-	1
*B*. *fragilis group*	-	-	100	-	-	-	25	-	7	-	-	132
*C*.*perfringens *	-	-	-	-	-	-	9	-	23	-	-	32
*C*.*difficile*	-	-	77	-	-	-	-	-	-	-	-	77
*Prevotella*	-	-	-	10	-	-	-	-	-	-	-	43
*Fusobacterium*	-	-	12	-	-	-	-	-	-	-		12
Total	264	64	26	44	14	-	260	49	99	40	-	1156

### Number of aerobic bacterial isolates from clinical specimens

In total, 497 GNB (57%) and 363 GPB (42%) were included in this study. The isolated GNBs were *E*. *coli* (n = 193/497; 38%), *Klebsiella* spp. (n = 97/497; 19%), *A*. *baumannii* (n = 95/497; 19%), *Enterobacter* spp. (n = 36/497; 0.02%), *P*. *aeruginosa* and *Proteus mirabilis* (n = 12/497; 0.02%), and *Citrobacter* spp. and *Stenotrophomonas* spp. (n = 1/497). Moreover, the main isolated GPBs included coagulase-negative *Staphylococcus* (CoNS; n = 130/363; 36%), *S*. *aureus* (n = 127/363; 34%), *Enterococcus* spp. (n = 32/363; 0.08%), *Stresptococcus* spp. (n = 62/363; 17%), and *Micrococcus* spp. (n = 12/363; 0.03%). Among GNBs and GPBs, *E*. *coli* and CoNS were the most common bacteria, respectively (Tables 3 and 4).

The article "Study of aerobic and anaerobic bacterial profile of nosocomial infections and their antibiotic resistance in a referral center, Southwest Iran: A three year cross-sectional study" was retracted in 2025. Reasons: lack of ethics approval or compliance; missing or withdrawn patient consent; concerns about the welfare of human subjects.

**Table 3:** The resistance rates of GNB to commonly used antimicrobials (2018–2020).

Gram-negative microorganisms																								
Antibiotics	*Acinetobacter* spp. (n = 95)			*Klebsiella* spp. (n = 97)			*E*. *coli* (n = 193)			*P*. *aeruginosa* (n = 62)			*P*. *mirabilis* (n = 12)			*Enterobacter* spp. (n = 36)			*Stenotrophomonas* spp. (n = 1)				*Citrobacter* spp. (n = 1)	
	2018	2019	2020	2018	2019	2020	2018	2019	2020	2018	2019	2020	2018	2019	2020	2018	2019	2020	2018	2019	2020	2018	2019	2020
AMK	15	45	35	10	33	52	55	35	101	10	27	25	3	3	6	6	15	15	NR*	NR	NR	-	-	1
AMP	S*	S	1	S	6	13	15	8	41	S	S	3	S	S	2	S	S	5	NR	NR	NR	-	-	-
CZO	1	3	1	7	17	17	15	15	45	1	2	2	S	S	S	S	S	5	NR	NR	NR	-	-	-
FEP	15	25	48	10	40	47	10	65	114	13	8	41	S	6	6	10	12	14	NR	NR	NR	-	-	1
FOX	NR	NR	NR	S	S	S	S	S	S	NR	NR	NR	S	S	S	S	S	S	NR	NR	NR	-	-	-
CRO	24	15	52	9	22	66	6	6	111	22	4	32	3	6	3	13	13	10	NR	NR	NR	-	-	1
CIP	17	30	45	15	31	45	38	22	116	17	15	30	S	6	5	8	7	18	NR	NR	NR	-	-	1
CLI	NR	NR	NR	NR	NR	NR	NR	NR	NR	NR	NR	NR	NR	NR	NR	NR	NR	NR	NR	NR	NR	NR	NR	NR
DOX	15	35	45	S	S	10	S	S	15	S	S	5	S	S	1	S	2	2	NR	NR	NR	-	-	-
ERY	NR	NR	NR	NR	NR	NR	NR	NR	NR	NR	NR	NR	NR	NR	NR	NR	NR	NR	NR	NR	NR	NR	NR	NR
GEN	8	8	2	3	3	10	10	10	14	S	6	6	S	1	2	S	S	6	NR	NR	NR	1	-	-
IMP	33	10	52	5	11	17	8	34	70	24	5	22	S	S	3	9	9	8	NR	NR	NR	1	-	-
NIT	NR	NR	NR	S	S	S	S	S	S	6	S	S	R	R	R	S	S	S	NR	NR	NR	-	-	-
PEN	NR	NR	NR	NR	NR	NR	NR	NR	NR	NR	NR	NR	NR	NR	NR	NR	NR	NR	NR	NR	NR	NR	NR	NR
TZP	5	15	16	S	S	6	S	S	6	S	23	30	S	S	1	S	S	1	NR	NR	NR	-	-	-
RIF	S	S	2	S	S	S	S	S	S	S	S	S	S	S	S	S	S	S	NR	NR	NR	-	-	-
TCY	7	36	22	10	6	39	15	55	57	2	10	22	S	2	2	S	4	6	NR	NR	NR	-	-	-
SXT	15	35	45	10	12	69	20	65	90	9	11	41	3	3	6	10	10	13	1	-	-	1	-	-
CAZ	9	36	37	11	25	16	20	32	33	5	5	15	S	5	5	S	7	18	1	-	-	1	-	-
SAM	S	29	52	6	3	3	S	S	15	S	S	S	S	S	S	S	6	3	NR	NR	NR	-	-	-
LEV	5	6	7	6	1	S	S	S	3	S	S	6	S	S	S	S	S	S	S	NR	-	-	-	-
MUP	3	5	6	3	S	S	S	S	S	S	S	S	S	S	S	S	S	1	NR	NR	NR	-	-	-
MNO	5	10	9	S	S	S	S	S	S	S	S	S	S	S	S	S	S	S	NR	NR	NR	-	-	-
LNZ	NR	NR	NR	NR	NR	NR	NR	NR	NR	NR	NR	NR	NR	NR	NR	NR	NR	NR	NR	NR	NR	NR	NR	NR
COL	S	S	S	S	S	S	S	S	S	1	1	11	S	S	S	S	S	S	NR	NR	NR	-	-	-
CCV	S	S	3	S	S	S	S	S	9	S	S	S	S	S	S	S	S	S	NR	NR	NR	-	-	-

**Abbreviations:** Ampicillin (AMP), Gentamicin (GEN), Ciprofloxacin (CIP), Ceftazidime (CAZ), Nitrofurantoin (NIT), Imipenem (IMI), Penicillin (PEN), Clindamycin (CLI), Erythromycin (ERY), Doxycycline (DOX), Trimethoprim/sulfamethoxazole (SXT), Colistin (COL), Linezolid (LNZ), Mupirocin (MUP), Rifampin (RIF), Amikacin (AMK), Ceftriaxone (CRO), Ceftazidime/Clavulanic acid (CCV), Minocycline (MNO), Cefazolin (CZO), Cefepime (FEP), Piperacillin /Tazobactam (TZP), Tetracycline (TCY), Ampicillin/Sulbactam (SAM), Levofloxacin (LEV), (NR*) = non-recombinant, (S) = susceptible.

The article "Study of aerobic and anaerobic bacterial profile of nosocomial infections and their antibiotic resistance in a referral center, Southwest Iran: A three year cross-sectional study" was retracted in 2025. Reasons: lack of ethics approval or compliance; missing or withdrawn patient consent; concerns about the welfare of human subjects.

**Table 4:** The resistance rates of GPB to commonly used antimicrobials (2018–2020).

Gram-negative microorganisms															
Antibiotics	*S*. *aureus* (n = 127)			*Enterococcus* spp. (n = 32)			*Micrococcus* spp. (n = 120)			*Streptococcus* spp. (n = 62)			*CoNS* (n = 130)		
	2018	2019	2020	2018	2019	2020	2018	2019	2020	2018	2019	2020	2018	2010	2020
AMK	22	50	55	7	12	13	4	2	6	S	4	3	30	25	72
AMP	S	3	3	6	5	20	S	S	1	S	4	2	S	S	2
CZO	S	1	2	S	1	2	S	S	S	S	S	S	S	2	4
FEP	S	S	S	S	S	S	S	S	S	S	S	S	S	S	S
CTX	S	S	S	S	S	S	S	S	S	S	S	S	S	S	S
FOX	42	18	59	S	S	2	S	S	7	S	S	S	23	35	69
CRO	S	S	2	7	5	19	S	S	S	S	S	S	S	S	S
CIP	46	33	43	S	S	S	1	S	1	S	2	5	26	42	47
CLI	37	21	69	NR	NR	NR	4	2	6	S	S	S	10	42	68
DOX	7	16	7	10	10	10	S	S	1	S	S	S	24	62	44
ERY	38	19	70	NR	NR	NR	4	4	4	S	2	5	44	22	64
GEN	S	S	4	S	S	1	2	2	6	S	S	S	S	2	2
IMP	68	10	36	14	5	10	4	2	6	S	2	5	41	22	58
NIT	S	S	2	S	S	S	S	S	S	S	S	S	S	S	S
PEN	13	44	54	4	12	15	4	3	5	5	S	2	27	42	38
TZP	S	S	S	S	S	S	S	S	S	S	S	S	S	S	S
RIF	S	S	6	S	S	S	S	S	S	S	S	S	S	S	S
TCY	21	30	20	S	4	4	4	2	6	S	4	1	19	20	38
SXT	42	33	47	10	11	10	4	2	6	S	5	2	44	22	58
VAN	29	22	13	10	10	12	4	2	6	S	4	2	19	24	20
BAC	S	S	2	S	S	1	-	-	7	S	S	S	7	12	18
CAZ	S	S	2	S	S	1	S	S	S	S	S	S	S	S	S
SAM	S	S	S	S	S	1	S	S	S	S	S	S	S	S	S
TEC	S	S	12	S	S	S	S	S	S	S	S	S	S	2	1
LEV	S	S	4	S	S	1	S	S	S	S	S	S	S	S	1
MUP	S	S	1	S	S	1	S	S	S	S	S	S	S	S	S
MNO	S	S	S	S	S	1	S	S	S	S	S	S	S	S	S
LNZ	S	4	6	S	S	1	S	S	S	S	S	S	S	S	S
COL	NR	NR	NR	NR	NR	NR	NR	NR	NR	NR	NR	NR	NR	NR	NR
CCV	S	S	2	S	S	S	S	S	S	S	S	S	S	S	S

Ampicillin (AMP), Gentamicin (GEN), Ciprofloxacin (CIP), Vancomycin (VAN), Ceftazidime (CAZ), Nitrofurantoin (NIT), Imipenem (IMI), Penicillin (PEN), Clindamycin (CLI), Erythromycin (ERY), Doxycycline (DOX), Trimethoprim/sulfamethoxazole (SXT), Colistin (COL), Linezolid (LNZ), Mupirocin (MUP), Rifampin (RIF), Amikacin (AMK), Ceftriaxone (CRO), Ceftazidime/Clavulanic acid (CCV), Minocycline (MNO), Cefazolin (CZO), Piperacillin/Tazobactam (TZP), Tetracycline (TCY), Ampicillin/Sulbactam (SAM), Teicoplanin (TEC), Levofloxacin, (LEV), Bacitracin (BAC), Cefoxitin (FOX), Cefotaxime (CTX), (NR*) = non-recombinant, (S) = susceptible.

### Number of anaerobic bacterial isolates from clinical specimens

Frequency of anaerobic bacteria were *B*. *fragilis* group (n = 132; 44%) followed by *Clostridium perfringens* (n = 32; 10%), *Prevotella* (n = 43; 25%), *Clostridium difficile* (n = 77; 26%), and *Fusobacterium* (n = 12; 4%).

### AMR rates of GNB to antimicrobials

Among GNBs, *P*. *aeruginosa* isolates were 100% resistant to amikacin, cefepime, ciprofloxacin, tetracycline, and nitrofurantoin. However, *P*. *aeruginosa* showed no level of resistance to levofloxacin, ciprofloxacin, and colistin. Ceftazidime/clavulanic acid and colistin were the most effective antibiotic against *A*. *baumannii*, minocycline, clindamycin, and colistin against *Klebsiella* spp., but against both *Enterobacter* spp. and *E*. *coli*, minocycline, clindamycin, nitrofurantoin, and colistin were resistant. Moreover, 100% resistance was observed for amikacin, doxycycline, trimethoprim-sulfamethoxazole, and imipenem. We also detected 100% resistance in *Klebsiella* spp. to cefepime and imipenem and also high resistance rate against amikacin and trimethoprim-sulfamethoxazole (n = 95/97; 97%). All *Enterobacter* spp. exhibited resistance to amikacin and ceftriaxone and a high level of resistance to trimethoprim-sulfamethoxazole (n = 33/36; 91%) and ceftazidime (n = 25/36; 69%). In case of *E*. *coli*, the resistance rate was very high (n = 191/193; 98%) for trimethoprim-sulfamethoxazole and cefepime. The resistance rates of each GNB to commonly used antimicrobials are represented in Table 3.

The article "Study of aerobic and anaerobic bacterial profile of nosocomial infections and their antibiotic resistance in a referral center, Southwest Iran: A three year cross-sectional study" was retracted in 2025. Reasons: lack of ethics approval or compliance; missing or withdrawn patient consent; concerns about the welfare of human subjects.

### AMR rates of GPB to antimicrobials

The resistance rates of GPB isolates to antimicrobial agents are illustrated in Table 2. In case of *S*. *aureus* isolates, the highest resistance rates belonged to amikacin and clindamycin (n = 127/127; 100% for both), followed by erythromycin (n = 64/127; 50%). However, *S*. *aureus* had the low levels of resistance to ampicillin/sulbactam. Trimethoprim-sulfamethoxazole and minocycline as well as linezolid and minocycline were the most efficient antimicrobials against *S*. *aureus* and CoNS, respectively. CoNS strains showed high-level resistance to doxycycline and erythromycin (n = 130/130; 100% for both) and cefoxitin (n = 127/130; 97%). The percentage distribution rates of methicillin-resistant *Staphylococcus aureus* (MRSA) and methicillin-resistant CoNS (MR-CoNS) were 93% (n = 119/127) and 97% (n = 127/130), respectively. *Enterococcus* spp. was 100% resistant to amikacin and ampicillin, and its resistance to ceftriaxone (n = 31/32; 96%), doxycycline, and erythromycin (n = 30/32; 93%) was also very high. However, *Enterococcus* spp. had low levels of resistance to linezolid and clindamycin. Detailed information on other GPBs is listed in Table 4.

### AMR rates of anaerobic to antimicrobials

The resistance rates of anaerobic isolates to antimicrobial agents are illustrated in Table 5. In case of *B*. *fragilis group* isolates, the highest resistance rates belonged to clindamycin (n = 96/132; 72%), followed by penicillin (n = 76/132; 57%). However, *B*. *fragilis group* had the low levels of resistance to metronidazole and imipenem were the most efficient antimicrobials against *fragilis group*. *C*. *perfringens* strains showed high-level resistance to penicillin (n = 20/43; 46%). The percentage distribution rates metronidazole resistant in *C*. *difficile* were 97% (n = 23/77;29%), respectively. The Table 5 shows the rest of the anaerobic bacteria and their antibiotic resistance.

The article "Study of aerobic and anaerobic bacterial profile of nosocomial infections and their antibiotic resistance in a referral center, Southwest Iran: A three year cross-sectional study" was retracted in 2025. Reasons: lack of ethics approval or compliance; missing or withdrawn patient consent; concerns about the welfare of human subjects.

**Table 5:** Antimicrobial susceptibility of anaerobic bacterial.

Agents	Penicillin	Cefoxitin	Chloramphenicol	Clindamycin	Metronidazole	Imipenem
	S* R*	S R	S R	S R	S R	S R
Bacterial Strains MCI (μg/mL)	≤ 0.5 ≥ 2	≤ 16 ≥ 64	≤ 8 ≥ 32	≤ 2 ≥ 8	≤ 8 ≥ 32	≤ 4 ≥ 16
B. fragilis group	36 96	100 32	109 23	76 56	109 23	122 10
*C*. *perfringens*	12 20	32 0	NR*	32 0	30 2	132 0
*C*.*difficile*	54 23	67 10	NR	65 12	54 23	NR
*Prevotella* spp	30 13	NR	NR	23 20	32 11	38 5
*Fusobacterium*. spp	12 0	NR	NR	12 0	12 0	12 0

*MIC, Minimal Inhibitory Concentration; (NR*) = non-recombinant; S, Susceptible; R, Resistant.

### Rates of MDR isolates

Overall MDR to all the isolates (n = 525/860) was 61%, 2018. 10% in 2019, 15% in 2020, and 36% in 2019. GNB *A*. *baumannii* (n = 95/95) had the highest MDR (100%), followed by *Klebsiella* spp. (n = 91/97; 93%), *E*. *coli* (n = 18/193; 0.09%), *Enterobacter* spp. (n = 3/36; 0.08%), *P*. *aeruginosa* (n = 12/62; 0.19%), and *P*. *mirabilis* (n = 12/62; 19%). The least MDR was identified in *Citrobacter* spp. and *Stenotrophomonas* spp. (n = 1/1; 100% for both; (Table 6). MDR of GPB *S*. *aureus* (n = 127/l27; 100%), *Micrococcus* spp. (n = 12/12; 100%), CoNS (127/130, 97%), and *Enterococcus* spp. (n = 29/32; 96%) was very high, but that of *Streptococcus* spp. (n = 7/62; 11%) was low (Table 7). No XDR and PDR isolates were detected in all the bacteria.

**Table 6:** The frequency of MDR in GNB.

	2018	2019	2020
***Acinetobacter* spp.**	16	22	57
***Klebsiella spp*.**	22	10	59
***E*. *coli***	3	4	11
***P*. *aeruginosa***	11	12	29
***P*. *mirabilis***	7	2	3
***Enterobacter* spp**	1	2	4
***Stenotrophomonas spp*.**	-	-	1
***Citrobacter* spp.**	-	-	-

**Table 7:** The frequency of MDR in GPB.

	2018	2019	2020
***S*. *aureus***	34	23	73
***Enterococcus spp*.**	13	10	6
***Micrococcus spp*.**	3	3	6
***Streptococcus spp*.**	21	12	29
***CoNS***	7	2	3

## Discussion

Uncontrolled use of antimicrobials for the treatment of infections has adverse effects on public health and results in drug resistance both in developed and developing countries. Thus, it is essential continuously evaluate the antimicrobial resistance condition in hospitals, which was the goal of the present study. To this end, the data of three consecutive years on antibiotic consumption in hospitals were recorded. In the current study, there was a relatively higher occurrence of the positive culture among samples collected from patients (n = 1156/1246; 92%) in comparison with other studies in Iran [17, 18]. This difference in the results may be due to the special climate of the southwest of Iran, which has humid and rather hot weather. In our study, similar to former surveys, *E*. *coli* and *Staphylococcus* were the most prevalent GNB and GPB, respectively [19, 20].

The article "Study of aerobic and anaerobic bacterial profile of nosocomial infections and their antibiotic resistance in a referral center, Southwest Iran: A three year cross-sectional study" was retracted in 2025. Reasons: lack of ethics approval or compliance; missing or withdrawn patient consent; concerns about the welfare of human subjects.

The present study evaluated the pattern of antimicrobial resistance among patients in the hospital by evaluating and comparing AMR condition in different years. According to the results, there was an increase in the presence of resistant bacteria among bacterial isolates in southwestern Iran from 2018 to 2020. Mihankhah *et al*. investigated the bacteria associated with urinary tract infection and antibiotic susceptibility profile of the isolates between 2013 and 2015 in the north of Iran. They found a great challenge of emerging multidrug-resistant strains of bacteria in Iran [21]. The results of other studies have also shown an increase in AMR [22–25]. Findings of the declining value of antibacterial mean that the treatment of patients is becoming difficult, costly, or even impossible. In low-income countries, extensive use of antibiotics is a common practice due to the high rates of both hospitalization and infectious diseases. On the other hand, the emergence of MDR bacteria is a challenge for physicians to manage critical patients. As noted, MRSA, extended-spectrum ß-lactamase (ESBL) *E*. *coli*, vancomycin-resistant *S*. *aureus*, and enterococcus-associated morbidity and mortality are global problems. Staphylococcus species, especially *S*. *aureus*, had the highest prevalence in our study (93%). The percentage distribution rates of MRSA and MR-CoNS were 93% (n = 119/127) and 97% (n = 127/130), respectively. It is worrying that *S*. *aureus* strains carrying resistance genes are isolated from various specimens. There are reports on *S*. *aureus* as a cause of disease in patients and on the increased prevalence of MDR isolates [26]. Comparable results were also obtained in another study, which showed the increase of MDR *S*. aureus strains. In contrast to our results, Savaş *et al*. reflected that only 24.1% of Staphylococci strains were isolated from patients [27].

This study suggested that Enterobacteriaceae family bacteria were the most common isolated GNB. In addition, *E*. *coli* was the most frequent pathogen, which is consistent with other studies [28, 29]. The results of antibiogram test for 497 bacterial isolates recovered from patients revealed that amikacin and imipenem were the most effective antimicrobials against the strains. Some GNBs, such as *Pseudomonas* and *Acinetobacter*, were resistant to these antibiotics, which are widely used for treating hospital-acquired infections. Carbapenems are resistant to β-lactamase enzymes produced by numerous MDR GNB, therefore playing a significant role in the treatment of infections not cured by other antibiotics. Hence, a probable increase of the imipenem-resistant strains can be an emerging concern for the health control systems of a country [30]. It seems that officials need to be more concerned about the use of these drugs for the treatment of infections. ESBL-producing organisms are capable of hydrolyzing penicillin, a broad spectrum of cephalosporins, and monobactams; however, they do not affect the cephamycins or carbapenems, and their activity is inhibited by clavulanic acid. Furthermore, ESBL-producing organisms often exhibit resistance to other antimicrobial classes [31]. We were able to find only suspicious ESBL isolates. In our study, eight *E*. *coli* and three *A*. *baumannii* isolates were suspected or talented ESBL producers in GNB. For a definitive diagnosis, phenotypic and genotypic methods are required. In the study performed by Abayneh *et al*., ESBL-producing phenotypes were detected in 23% of urinary isolates, of which *E*. *coli* accounts for 76.5% (n = 13) and *K*. *pneumoniae* for 23.5% [32]. AMR data for all three years of surveillance showed significant resistance of GNB (*A*. *baumannii*, *K*. *pneumonia*, and *P*. *aeruginosa*) and GPB (*S*. *aureus*, CoNS, and Micrococcus spp.) to many antibiotic classes. Our findings indicated that AMR has growth during the study period (from 2018 to 2020), and this elevation is a serious warning to hospitals, medical staff, and physicians. Based on the results, the rate of MDR bacteria elevated from 10% to 36%, and there is a possibility of a further increase in the coming years. Overall, 61% of isolates were MDR. In a similar study performed in the north of Iran, a remarkable rate of MDR isolates (62.8%) was found, which displayed an increasing trend [28]. The MDR prevalence in Asia is 50% [33], very high in Saudi Arabia [34], and 13% in India [35]. In the past, β-lactam antibacterial agents were often used to treat anaerobic infections. Now, anaerobes have shown a propensity for development of resistance to these agents. Seventy-two percent B. *fragilis* isolates were resistant to penicillin, which is similar to findings of other researches. In recent years, development of resistance of the *B*. *fragilis* group to cephalosporins has been distribution. In this study, 24% of *B*. *fragilis* isolates and 100% of *C*. *perfringens* isolates were susceptible to cefoxitin, respectively. In contrast, most of *B*. *fragilis* isolates were sensitive to clindamycin, chloramphenicol, metronidazole, and imipenem, respectively, which are in agreement to the results of other works [36, 37]. Given that the study shows an increasing trend of AMR, particularly the prevalence of isolates in the hospital, it is suggested that physicians be more careful in prescribing antibiotics to patients, and in future studies on physicians’ knowledge about isolates, a questionnaire is prepared. Certainly, providing more information to doctors and being more careful with the microbial department of the laboratory will reduce the trend of AMR in the future. There are limitations in our study, it would be better to use molecular methods to more accurately identify isolates.

The article "Study of aerobic and anaerobic bacterial profile of nosocomial infections and their antibiotic resistance in a referral center, Southwest Iran: A three year cross-sectional study" was retracted in 2025. Reasons: lack of ethics approval or compliance; missing or withdrawn patient consent; concerns about the welfare of human subjects.

## Conclusions

Although the eradication of AMR is impossible, effective planning and management might reduce its risks and negative consequences. Iran has formulated a nationwide action plan to combat AMR, which needs to be ratified. Nevertheless, the growing trend of AMR in the country in previous years has created a major challenge to the health system. The results highlighted that there are distinct and political factors leading to AMR in Ahvaz, a developing city of Iran. It may be due to the climate and nature of the southwest area of Ahvaz, which has humid and relatively hot weather. The primary contributors to the resistance development include the weak surveillance of drug-resistant infections, clinical misuse, and easy access to antibiotics. Moreover, similar factors such as self-medication and the lack of regulation on medication imports are responsible for AMR. It is important to have clear guidelines set by an international health agency, such as the WHO, to maintain consistency across nations. However, since each country has varied health care and regulatory system, its policies to manage antibiotic use are different. Besides, different aspects of the regulatory system would need to be further improved based on the specific challenges in each country.
